The article "Application of Psychological Contract Theory in Mental Health and Professional Development of University Teachers" was retracted in 2023. Reasons: signs of a paper mill; suspected computer-generated content; unreliable results or conclusions; concerns about the data.

# Application of Psychological Contract Theory in Mental Health and Professional Development of University Teachers

**DOI:** 10.1155/2022/6985766

**Published:** 2022-08-25

**Authors:** Huixiao Zhang

**Affiliations:** School of Foreign Languages, Hebei University of Science and Technology, Shijiazhuang, China

## Abstract

Mental health is an important element of human public health. To investigate the respective causes of and the relationship between effort-reward imbalance and psychological anxiety of university teachers, the author, after making a targeted survey of more than 2000 questionnaires and conducting statistics and analysis of the survey data, discovers that the effort-reward imbalance has a significant effect on the anxiety of university teachers and meanwhile, effort-reward imbalance will indirectly affect the anxiety of university teachers through the breach of psychological contracts and thus directly affect the mental health of university teachers. To solve this problem, the author takes advantage of the psychological contract theory and designs a mental health improvement system for university teachers, that is, to pay more attention to the feeling of effort-reward balance of young university teachers, to give more care and help to teachers who have imbalance feelings, to take the maintenance of psychological contracts as an important starting point of the ideological work of young teachers in universities, and so on. Through the implementation of relevant systems, colleges and universities have effectively strengthened their ability to fulfill contracts, established convenient and unobstructed communication channels, prevented breach of psychological contracts of teachers, and prevented teachers from working at high exhaustion at the cost of their physical and mental health, which can finally improve the job satisfaction and professional development of university teachers and enable them to be devoted to higher education in better health.

## 1. Introduction

The healthy psychology of teachers has positive effects on students' emotion, personality, motivation, and other psychological factors and can also benefit teachers' own career development, physical and mental health, and happiness in life [1]. As an important part of mental health education, psychology of teachers has attracted extensive attention of researchers. After decades of exploration, the research on psychology of teachers in China has made breakthroughs both in depth and in breadth. It is of great theoretical value and practical significance to understand the current situation, pay attention to the hot spots, and reflect on the existing problems of research on psychology of teachers for promoting research on psychology of teachers in China, improving the level of teachers' mental health and enhancing the mental health education ability of schools. An Fuhai analyzed the hot spots and developing trend of the research on psychology of teachers in China in the past 20 years by using CiteSpace, an information visualization software, and the results show that the hot spots include teachers' psychological characteristics and psychological contract, and psychological contract has become an important factor of teachers' mental health in colleges and universities [2]. The administrators of colleges and universities have also taken many measures to maintain the relative stability of the teaching staff, such as signing documentary contracts, raising salary and welfare, and formulating various preferential policies; however, it cannot stop the leaving of some prominent teachers [3–6]. Some administrators also propose to “retain staff by improving treatments and through emotions,” but with only inconspicuous effects for lack of scientific instructions of operation [7–10]. Therefore, in college and university teaching staff management, besides applying the management method of “documentary contracts,” we cannot ignore the effect of “psychological contracts.” Deriving from psychological theories of the US, “psychological contract” theory is employed in this paper to analyze the stable development of college and university teaching staff [11–14].

The article "Application of Psychological Contract Theory in Mental Health and Professional Development of University Teachers" was retracted in 2023. Reasons: signs of a paper mill; suspected computer-generated content; unreliable results or conclusions; concerns about the data.

## 2. Connotation and Characteristics of “Psychological Contract” Theory

“Psychological contract” is a phrase first put forward by Professor Argyris, a famous organizational psychologist in the US, which was later completed by Levinson and other scholars. He thought that psychological contract was a match between what the individual will give and what the organization desires to gain and what the organization will provide in response and what the individual expects to gain. The study on psychological contract is a hot topic emerging in human resources, organizational behavior, psychology, and other domains. Along with the arrival of the era of knowledge-driven economy, some contradictions in labor relations stand out under the effect of the global environment such as organizational adjustment of schools (e.g., strategic target up-moving, business outsourcing, pyramid structure flattening, etc.), staff redundancy, and organizational reform because of the globalization of competition. Harmonious labor relations are the basis for a harmonious society, and the construction of harmonious labor relations becomes one of the important topics in society nowadays. British psychologists think that during the organizational structure adjustment of schools and the alteration of employment relationships, psychological contract is the most sensitive core factor that can reflect such change in the most concentrative way. Many experts in organizational behavior think that psychological contracts have important influence on the attitude and behavior of the individuals in the organization. The study on psychological contracts in organizations can be an effective way to adjust and control organizational behavior, enhance organization efficiency, improve teachers' satisfaction, and construct harmonious labor relations [15–18]. Besides expressly stipulated provisions, there are some invisible expectations in various contractual relationships in colleges and universities. For instance, students care whether the knowledge learned is equivalent to the expenditure, teachers care about the relevancy between what they give and what they get, and schools pay attention to the input-output ratio; therefore, there are some psychological contracts among colleges and universities and teachers and students. Hence, this paper thinks that, in colleges and universities, psychological contract means through mutual psychological-level implications and perceptions between schools and teachers, responsible organizations of colleges and universities inspire teachers' external motivation to teaching development, satisfy teachers' individual expectations, and establish a complete mechanism and agreement of invisible rights and obligations [19–22].

The article "Application of Psychological Contract Theory in Mental Health and Professional Development of University Teachers" was retracted in 2023. Reasons: signs of a paper mill; suspected computer-generated content; unreliable results or conclusions; concerns about the data.

## 3. Research Status and Related Theories of Psychological Contract Theory

With the deepening of the reform of the employment and assessment system in colleges and universities, the survival and development anxiety felt by young university teachers increases day by day [3]. Some studies believe that, in addition to the pressure from work and life, one direct cause of anxiety of young university teachers is the imbalanced feeling of high efforts and low rewards they experience [10]. According to the effort-reward imbalance theory proposed by Siegrist [23], individual stress response at work is not only related to task load and role requirements, but also related to the effort-reward feelings in completing tasks. When the time, energy, and emotion invested in work are not equally reciprocated (effort-reward imbalance), this will cause negative emotional and behavioral consequences for the individual. From the perspective of social exchange, Siegrist pointed out that the effort-reward imbalance, as a kind of exchange failure, would cause persistent and strong stress response of the individual and damage individual health through specific neural response systems. However, Siegrist did not strictly distinguish the effect difference of internal and external efforts at that time. Instead, he took external factors such as job responsibilities, time pressure, and task requirements as the main contents of efforts. In the subsequent application of the model, Siegrist et al. gradually separated the state of overcommitment, representing individual overimmersion in work, from the original effort factors, and pointed out that overcommitment would exacerbate the negative impact of effort-reward imbalance on individual health [23–25].

The article "Application of Psychological Contract Theory in Mental Health and Professional Development of University Teachers" was retracted in 2023. Reasons: signs of a paper mill; suspected computer-generated content; unreliable results or conclusions; concerns about the data.

The typical aftereffect of effort-reward imbalance is the impact on individual emotional health. According to the emotional cognitive evaluation theory, when faced with stress stimulus, the individual will first evaluate the impact of the stimulus before triggering specific emotional responses. It means that there may be a very important relationship between effort-reward imbalance and the anxiety of young university teachers. A direct reaction of effort-reward imbalance is an evaluation of the reciprocal relationship by the individual between himself and the organization, that is, to judge whether the organization has equally performed the commitment of matching efforts and rewards. The individual perception of the organization's performance of commitment is also called the psychological contract, which refers to the individual feeling of whether his psychological expectation of the organization's fulfillment of obligations and responsibilities has been satisfied. If young teachers feel that the school fails to perform the due commitment, they will consider that the school has violated the reciprocal agreement, and this will lead to the breach of the teachers' psychological contract, weaken teachers' predictability and sense of control at work, cause unsafe work feelings of teachers, and eventually cause teachers' anxiety. Meanwhile, according to the effort-reward imbalance theory, the breach of psychological contracts also reflects the imbalanced employment relationship between teachers and schools, which, as a typical source of social psychological pressure at work, will easily lead to anxiety among teachers. Recent studies on firefighters have also shown that breach of psychological contracts can significantly predict individual anxiety and depression. Therefore, it is speculated that psychological contract breach may play an intermediary role in the relationship between effort-reward imbalance and anxiety. Overcommitment is a key factor affecting the aftereffect of effort-reward imbalance. It refers to the attitudinal, behavioral, and emotional characteristics of overimmersion in work of individuals driven by a strong desire to be recognized and respected. Teachers with high overcommitment devote more emotion and energy to their work and have a stronger desire to be recognized and respected, so they may be more sensitive to efforts and rewards, while teachers with low overcommitment consume less emotion and energy in their work and have lower expectation and sensitivity to rewards. Therefore, colleges and universities should design and establish a perfect teacher management system under the guidance of psychological contract theory to clarify the responsibilities and expectations of both sides so as to improve the mental health of university teachers [11, 26–34].

The article "Application of Psychological Contract Theory in Mental Health and Professional Development of University Teachers" was retracted in 2023. Reasons: signs of a paper mill; suspected computer-generated content; unreliable results or conclusions; concerns about the data.

## 4. Investigation and Analysis on Effort-Reward Imbalance and Anxiety of University Teachers

### 4.1. Sample Extraction

The cluster sampling method is adopted this time to conduct an online survey on university teachers from 5 provinces of China, with 3,240 questionnaires collected in total and after removing samples with abnormal data, 3,125 valid samples are collected as follows:

1. Gender: male 52.8%, female 47.2%
2. Discipline: science and engineering 61.9%, literature and history 39.1%
3. Professional title: senior titles 22.1%, intermediate titles 53.2%, and junior titles 24.7%
4. Seniority: 3 years or below 29.3%, 4–6 years 41.3%, 7–9 years 20.3%, and 10 years or above 9.1%

Therefore, the samples are evenly distributed and strongly representative. Three methods including the effort-reward imbalance and overcommitment scale are used in the survey as follows.

#### 4.1.1. Effort-Reward Imbalance and Overcommitment Scale

Li Xiuyang's method is adopted for measurement, where the effort-reward subscale adopts a 5-point scale, and the higher the score, the higher the level of efforts and rewards; the overcommitment scale adopts a 4-point scale, and the higher the score, the higher the degree of individual overimmersion in work. The formula adopted is as follows:

(1) $$\begin{array}{c} \text{ERI}=\frac{E}{R}, \end{array}$$

where ERI is effort-reward ratio, *E* is average score of efforts, and *R* is average score of rewards. ERI > 1 indicates effort-reward imbalance.

#### 4.1.2. Psychological Contract Breach Scale

The psychological contract breach scale proposed by Shen Yimo et al. is adopted based on a 5-point scale. The higher the score, the higher the degree of psychological contract breach felt by the individual.

#### 4.1.3. Anxiety Self-Rating Scale

The method proposed by Wang Xiangdong et al. is adopted based on a 4-point scale. The higher the score, the higher the degree of the anxiety felt by the individual.

### 4.2. Result Statistics

The common method bias is controlled both in advance and afterwards and the analysis shows that the common bias is within a reasonable range and there is no multicollinearity problem. It can be seen from Table 1 that the average effort-reward ratio of university teachers is 1.36, indicating the effort-reward imbalance state of university teachers, and the average value of anxiety of university teachers is 2.95, indicating the relatively high anxiety level of university teachers. Meanwhile, it also shows that the effort-reward imbalance is significantly positively correlated with anxiety and psychological contract breach, and psychological contract breach is also significantly positively correlated with anxiety.

The article "Application of Psychological Contract Theory in Mental Health and Professional Development of University Teachers" was retracted in 2023. Reasons: signs of a paper mill; suspected computer-generated content; unreliable results or conclusions; concerns about the data.

The intermediary effect of psychological contract breach is tested as shown in Table 2. Effort-reward imbalance has a significant positive prediction effect on psychological contract breach, and psychological contract breach has a significant positive prediction effect on anxiety. Bootstrap analysis results of bias correction show that the intermediary effect of psychological contract breach on the relationship between effort-reward imbalance and anxiety is 0.09 (accounting for 28.22%), which reaches a significant level. Since the direct effect of the effort-reward imbalance on anxiety reaches a significant level (95% CI), psychological contract breach has an intermediary effect to some extent.

### 4.3. Statistical Analysis

University teachers do have the feeling of effort-reward imbalance, and their anxiety is at a relatively high level. Furthermore, young university teachers make a low evaluation of their sense of gain in their current career and feel anxious about it. Statistics show that effort-reward imbalance will cause anxiety not only directly, but also indirectly through psychological contract breach. The feeling of effort-reward balance is an important factor affecting the emotional state of university teachers. Effort-reward imbalance also indicates the thought of university teachers that they are “unfairly treated,” believing that the school fails to provide the feedback and support they deserve, which breaks the basic idea of reciprocity and thus causes them negative feelings like “contract breach.” As for the moderating effect of overcommitment, according to the social exchange equity theory, the reciprocal relationship between teachers and colleges and universities is also based on the equivalence of cost and return, and exchange equivalence not only refers to the equivalence of external benefits, but also includes the equivalence of internal emotions. When faced with effort-reward imbalance, teachers with high overcommitment will think that they have not established an equal exchange relationship with the school and their “excessive efforts” are not recognized by the school, which exacerbates psychological contract breach of the individual. The administrators of colleges and universities have also taken many measures to maintain the relative stability of the teaching staff, such as signing documentary contracts, raising salary and welfare, and formulating various preferential policies; however, it still cannot stop the leaving of some prominent teachers. Some administrators also propose to “retain staff by improving treatments and through emotions,” but with only inconspicuous effects for lack of scientific instructions of operation. Therefore, in college and university teaching staff management, we should make the utmost of the effect of “psychological contracts.” It is necessary not only to encourage and protect young teachers' aspirations to forge ahead and devote themselves to teaching and scientific research, but also to prevent teachers from working at high exhaustion at the cost of their physical and mental health. In the meantime, it is also necessary to guide university teachers to establish a correct view of gain and loss and enhance their ability to coordinate work and life so as to enable them to be devoted to higher education in better health.

The article "Application of Psychological Contract Theory in Mental Health and Professional Development of University Teachers" was retracted in 2023. Reasons: signs of a paper mill; suspected computer-generated content; unreliable results or conclusions; concerns about the data.

## 5. Performance of Psychological Contracts of University Teachers

### 5.1. Formation of Psychological Contracts

According to the characteristics of school management and elements of contracts, the performance of college and university teaching development psychological contracts include the satisfaction of three aspects, namely, school expectations, teacher expectations, and student expectations. The development of schools can be deemed as “Two Points, One Line.” The two points refer to students and teachers and the one line refers to the school. It means that the development of students and teachers and the formulation and implementation of school policies supplement each other. On the other hand, schools expect teachers to have good teaching motives and the demand of “I want to develop,” which guarantees the performance of teacher responsibilities; meanwhile, schools also expect students to have good learning motives and the pursuit of “I want to learn” so as to guarantee the performance of student responsibilities. In accordance with the system theory, schools can only develop continuously when teachers and students perform their responsibilities simultaneously. However in this system, student learning motives depend to a large extent on the “teaching charms” and “teaching arts” of teachers besides self-demand; meanwhile, teachers urgently expect the supportive behaviors (teaching instructions) of schools, and teachers can only generate the attitude and behavior of “I want to develop” when they perceive that schools are performing their responsibilities seriously; and at the same time, teachers also expect students to have strong learning motives to guarantee the performance of student responsibilities. Therefore, teacher satisfaction can only be realized when schools and students perform their responsibilities simultaneously; teachers' psychological contract of teaching development only takes shape when schools and teachers are both satisfied and when they perceive that the actual performance of responsibilities and obligations of the other conforms to their expectations.

The article "Application of Psychological Contract Theory in Mental Health and Professional Development of University Teachers" was retracted in 2023. Reasons: signs of a paper mill; suspected computer-generated content; unreliable results or conclusions; concerns about the data.

### 5.2. Establishment of Psychological Contracts

The establishment of psychological contracts of university teachers starts when young teachers enter their positions. Maslow once proposed the five-level model of human needs, the hierarchical structure of which being the motivation theories in psychology. The five-level model of human needs is usually described as levels in a pyramid. From the bottom of the hierarchy up, the needs are physiology (food and clothing), safety (job security), social needs (friendship), esteem, and self-actualization. Such five-hierarchy model can be divided as insufficiency needs and development needs. Maslow pointed out in 1943 that people needed motives to realize some needs and some needs shall be satisfied before others. For young teachers, they constantly pursue their goals and hope to satisfy Maslow's “five basic human needs” to different extents through their unremitting efforts. For this purpose, schools create platforms for the development of every teacher through competitions, such as “young teachers' lecture contest,” “multimedia courseware writing contest,” and “teachers' innovation contest”; schools provide opportunities for experimental learning in industries to improve teachers' practical ability and opportunities for further study through academic visits at home and abroad, attending academic conferences at home and abroad and advanced studies in elite schools. Therefore, in the establishment stage of psychological contracts, young teachers' career can develop rapidly and healthily, which can avoid the violation of psychological contracts.

### 5.3. Violation and Breach of Psychological Contracts

The violation and breach of psychological contracts means that when the expectations of both parties are not satisfied, psychological discrepancy will occur. It is also the perception and evaluation of one party of the contract that the other party fails to perform his due responsibilities and obligations in the psychological contract. The breach of psychological contracts is closely linked to the commitments of schools and the implementation of commitments, and it usually relates to psychological expectations of social benefits, development space, and embodiment of self-value. In colleges and universities, the violation and breach of psychological contracts means that teachers, after performing their teaching responsibilities, perceive that schools fail to perform or fail to perform in a proactive way their behaviors to support teachers' teaching development and then generate emotions or behaviors, such as working slow, job burnout, and even demission, which lead to the termination of psychological contracts.

The article "Application of Psychological Contract Theory in Mental Health and Professional Development of University Teachers" was retracted in 2023. Reasons: signs of a paper mill; suspected computer-generated content; unreliable results or conclusions; concerns about the data.

### 5.4. Adjustment and Remedy of Psychological Contracts

As described above, schools, teachers, and students can only be correspondingly satisfied and then further maintain the psychological contract when they perform their responsibilities simultaneously and their expectations are met; otherwise, psychological contracts will be violated and breached. As for teachers, their psychological characteristics and expectations will change along with the growing of their age and the changing of the environment, and school organizations also have different development demands in different periods and in different development stages. It can be seen that psychological contracts are not unchangeable but “dynamic,” which require both parties to the contract to conduct necessary adjustments in their interaction which may or may not meet the expectations and the expectations after adjustment cannot always be perceived by the other party in time. When the expectation of one party is not satisfied, there is a possibility of breach of psychological contracts; and the remedial measures taken by both parties when they sense breach or possibility of breach are the remedies of the psychological contract. If the remedial measures are rational and meet the expectations of both parties, they continue to perform their responsibilities and obligations and thus to complete the remedy of psychological contracts. During the whole reparative process, the attitude and behaviors of the school play a vital role.

## 6. Establishment of Favorable Psychological Contract System between Schools and Teachers and Promotion of Teachers' Mental Health

### 6.1. Establishing Perfect New-Teacher Training System to Strengthen Mutual Acceptance

In the early stage after new teachers enter schools, they feel fresh to study and work and take an active attitude. Schools are expected to provide them with sound interpersonal environment, respect and recognition, humanistic care, and opportunities of training and promotion. Study shows that teachers' subjective feelings to organizations and work influence the state of teachers' psychological contract to a large extent. Expectations of new teachers may differ from reality; that is to say, teachers are in the collision stage with organizations and organizations need to help teachers get rid of previous assumptions and replace them with another set of expectations admitted by the organization.

The article "Application of Psychological Contract Theory in Mental Health and Professional Development of University Teachers" was retracted in 2023. Reasons: signs of a paper mill; suspected computer-generated content; unreliable results or conclusions; concerns about the data.

New-teacher induction training is the “dashpot' of the collision stage. Induction training not only inculcates the values and ideas of the organization; rather, it leads new teachers to understand and then accept the criterion and values of the organization. The content and manner of induction training should be decided according to the education background, age, and experience of new teachers as well as the characteristics of the position. The training should mainly focus on pre-job guiding training (e.g., introductions to the school environment, work flow, working relationship, and school culture) aiming at job requirements. The aim of the training is to help new teachers to adapt to the environment of the school and integrate to the school as well as to enhance their sense of belonging to the school. In addition, induction training can help new teachers to coordinate interpersonal relationships, overcome their inadaptation to the job due to knowledge or experience, reduce working pressure, and narrow the gap between ideal and reality. Training can reduce the negative influence of internal and external factors to teachers and help teachers to form accurate role expectation to the school. For the same organization, it can employ the same mode but not necessarily the same content for new-teacher training. To eliminate new teachers' sense of unfamiliarity to the working environment and help them understand the practical work flow, they can go in classrooms to view and emulate the teaching process of aged teachers and aged teachers can make demonstrations and explanations for them. In order to help new teachers to get familiar to the environment and integrate into the new group, schools can arrange prominent or model teachers to have informal discussions with new teachers, answer their questions, and design phased targets for them. Prominent or model teachers should at the same time pass on experiences and lessons to new teachers to avoid their unrealistic expectations to work achievements. Besides, providing specific career planning and setting concrete job targets for new teachers are also important links to mitigate psychological shock.

The article "Application of Psychological Contract Theory in Mental Health and Professional Development of University Teachers" was retracted in 2023. Reasons: signs of a paper mill; suspected computer-generated content; unreliable results or conclusions; concerns about the data.

### 6.2. Establishing Sound Bilateral Relationships and Clearly Defining Responsibilities and Expectations of Both Parties

Psychological contracts determine teachers' behavior to the school to a certain extent; therefore, it is of great necessity for administrators of colleges and universities to understand the content of teachers' psychological contracts. At the same time, it is also of great importance for teachers to understand the decision of school administrators. Therefore, they should enhance mutual exchange and communication. Schools should explain their decisions to teachers in time so that they can understand the long- and short-term goals of development of the school. Before making decisions of major reforms, schools should listen to the opinions of teachers extensively and explain to teachers to get their support and understanding after making decisions. In times of difficulties when schools fail to realize partial of their commitments and responsibilities, they should explain to teachers to the greatest extent to get their understanding. Meanwhile, schools should try to know the psychological expectation of every teacher to the organization and increase emotional involvement in many ways, such as conferences, questionnaires, and trade union activities. When their expectations are satisfied, teachers can burden more psychological responsibilities and fulfill more obligations. When the psychological agreement of teachers to organizations is basically the same in content with the psychological agreement of organizations to teachers, the work efficiency of teachers can be improved and the psychological contracts can be maintained. So, schools should care more about the staff and every member should clearly know his position, responsibilities, rights, and obligations in the organization. As for young and middle-aged teachers, the organization should help them get the sense of achievement as soon as possible and let them know that the school sincerely cares about them and helps them with their development. As for aged teachers, the school should also let them know the expectations from them in school development through various ways and let them recognize that their development coexists with the development of the school and they can only realize their value by integrating their development in the development of the school.

### 6.3. Providing Fair Competition Environment and Development Space

One of the essential conditions to maintain the psychological contract between teachers and organizations is fairness and justice. The formulation of policies of stimulations and expectations from teachers should be fair, and the executive procedure should be just so that teachers will not feel discriminated or unfairly treated. When they cannot feel the expectation and stimulation of the organization, their expectations from the organization will reduce and they will show no more commitment to responsibilities or obligations. When teachers shoulder more responsibilities and obligations, the organization should response accordingly in time so that teachers can maintain their psychological balance, constantly adjust the content of the psychological contracts, actively maintain the psychological contracts, feel the expectation of the school to every hardworking teacher and feel that they can realize their value as long as they strive. Salaries and welfares are important goals of teachers' work and they should be in direct proportion to teachers' work. Teachers with higher salaries and better welfares should shoulder more tasks and bigger responsibilities. The two parties of the “psychological contract” are psychologically equal, and the instructions of administrators can only be put into practice consciously by teachers when they accept them actively and voluntarily rather than passively. In interpersonal relationships, administrators cannot blindly ask the subordinate to obey. They should try to create a common psychological basis and erect common objectives of the struggle so that the staff can obtain the sense of belonging, give full play to their advantages and potentials, get job satisfaction, realize their value to the development of the school, generate strong motives, show proactive working behaviors, and stay loyal to the organization.

The article "Application of Psychological Contract Theory in Mental Health and Professional Development of University Teachers" was retracted in 2023. Reasons: signs of a paper mill; suspected computer-generated content; unreliable results or conclusions; concerns about the data.

### 6.4. Providing Hierarchical Guidance and Planning Teachers' Career Scientifically

Teachers' career planning is the imagination and planning of every stage of teachers' career development. Teachers will have different psychological characteristics and expectations in different stages of development as they age, and these psychological changes will certainly influence their career development. By combining the comments of scholars both at home and abroad, we can divide teachers' career development into the early stage of entry, mid-career stage, and late-career stage. In the early stage of entry, new teachers have high work enthusiasm and strong demand for teaching development. During this period, the school only needs to design training programs scientifically, and teachers will actively cooperate and participate in them proactively. In the mid-career stage, the teaching process gradually becomes a production line for teachers. Schools can encourage teachers by establishing the teacher development assessment system, advocating “high quality and excellent teaching,” and adopting exceptional employment and preferential employment so as to promote teachers' teaching development. During this period, textual contracts play a decisive role. In the late-career stage, most teachers may suffer from job burnout. Schools can actively create conditions to show the charisma of aged teachers and give full play to their role of “passing, helping, and leading” so that they can feel their own value and at the same time do more teaching responsibilities. During this period, psychological contracts play a leading role in teachers' teaching development.

The article "Application of Psychological Contract Theory in Mental Health and Professional Development of University Teachers" was retracted in 2023. Reasons: signs of a paper mill; suspected computer-generated content; unreliable results or conclusions; concerns about the data.

### 6.5. Emphasizing Loving Care and Promoting Development of Teachers

Many researchers have conducted repeated surveys of different teachers and conclude that most teachers think that “they owe less to the organization while the organization owes more to them.” For new teachers, the organization should provide them with education about organizational socialization and improve their sense of ownership. Teachers should know that they are interdependent with the school and can not always passively wait for the school to realize their expectations. Sometimes they can take the initiative to let administrators of the organization understand their expectations and commitments of responsibilities and obligations. In psychological contracts, both parties construct psychological contracts based on perceptions of the other's work performance. Only when the administrators see your contribution to the school will they value you more, have positive expectations for you, show more commitments of the organization to you, and give you more conditions for your satisfaction and development. Therefore, both organizations and teachers should abandon some psychological contracts that cannot be realized according to the reality. They will create unrealistic expectations and promises that are not guaranteed to be fulfilled, leading to lower work ethics and higher demission rate among new teachers.

## 7. Experiment

Relevant experiment was carried out in a pilot university, and a questionnaire survey was conducted half a year later. The statistics are as follows:

1. *Degree of Satisfaction with the System*
2. Male teachers—82.5%, female teachers—86.7%
3. Young teachers—87.6%, middle-aged and elderly teachers—79.8%
4. Senior-title teachers—83.2%, intermediate-title teachers—85.6%, and junior-title teachers—87.9%
5. *Degree of Improvement of Teacher Satisfaction Compared with the Past*
6. Male teachers—15.7%, female teachers—16.2%
7. Young teachers—19.8%, middle-aged and elderly teachers—13.6%
8. Senior-title teachers—12.3%, intermediate-title teachers—15.7%, and junior-title teachers—17.8%

It can be seen that most teachers are satisfied with the implementation of the system and the mental health improvement system for teachers based on the psychological contract theory is successful.

The article "Application of Psychological Contract Theory in Mental Health and Professional Development of University Teachers" was retracted in 2023. Reasons: signs of a paper mill; suspected computer-generated content; unreliable results or conclusions; concerns about the data.

## 8. Conclusion

The mental health of teachers is the cornerstone to ensure the steady improvement of teaching quality and teaching order in colleges and universities. After 20 years of development, the content of teachers' psychological contract in China is more diversified and distinctive, and the maintenance mechanism of psychological contracts is becoming more complete and more targeted. This paper explores the potential effect mechanism of effort-reward imbalance on university teachers' anxiety through psychological contract breach and proposes the boundary conditions of the effect of effort-reward imbalance on anxiety. To better solve this problem, firstly, it is necessary to pay more attention to the feeling of effort-reward balance of young university teachers and give more care and help to teachers who have imbalance feelings in order to relieve teachers' anxiety caused by feeling of imbalance; secondly, it is necessary to take the maintenance of psychological contract as an important starting point of the ideological work of young university teachers, strengthen the ability of colleges and universities to fulfill contracts, and establish a convenient and unobstructed communication channel to prevent psychological contract breach of teachers; furthermore, we should develop a correct view on overcommitment of young university teachers at work. It is necessary not only to encourage and protect young teachers' aspirations to forge ahead and devote themselves to teaching and scientific research, but also to prevent teachers from working at high exhaustion at the cost of their physical and mental health. In the meantime, it is also necessary to guide young university teachers to establish a correct view of gain and loss and enhance their ability to coordinate work and life so as to enable them to be devoted to higher education in better health. Based on psychological contract theory, this paper establishes a favorable psychological contract system between schools and teachers and builds a more complete maintenance mechanism of teachers' psychological contract so as to enhance teachers' job satisfaction and happiness, improve teachers' mental health, and promote the continuous improvement of education quality in China.

## Figures and Tables

**Table 1:** Descriptive statistical results of variables.

	Variable	M	SD
1	Effort-reward imbalance ratio	1.36	0.49
2	Psychological contract breach	3.76	1.15
3	Overcommitment	2.91	0.55
4	Anxiety	2.95	0.53

**Table 2:** Test results of the intermediary effect of psychological contract breach.

Independent variable	PCB			AN		
	*β*	SE	*t*	*β*	SE	*t*
Gender	0.05	0.19	0.07	−0.03	−0.07	−0.23
Age	0.04	0.16	0.07	0.08	0.10	0.32
Seniority	−0.05	0.12	−0.05	0.07	0.12	0.45
Professional title	0.12	0.16	0.68	0.08	0.17	0.48
ERI	0.27	0.06	4.65	0.20	0.06	3.05
*R* ^2^		0.39			0.46	
*F*		10.52			13.32	

Indirect effect	Effect value		SE		95% CI	
	0.09		0.06		(0.045, 0.192)	
Direct effect	0.21		0.09		(0.134, 0.296)	

The article "Application of Psychological Contract Theory in Mental Health and Professional Development of University Teachers" was retracted in 2023. Reasons: signs of a paper mill; suspected computer-generated content; unreliable results or conclusions; concerns about the data.

## Data Availability

All the data contained in this study can be obtained from the corresponding author upon request and within the article.

## References

[1] Yu G. L., Zeng P. P. (2001). Teacher’s mental health and its improvememt. *Journal of Beijing Normal University*.

[2] An F. H., Zhao H. Y. (2022). 20 Years of research on teacher psychology in China:progress and reflection—an visual analysis based on CiteSpace knowledge map. *Theory and Practice of Education*.

[3] Yang J. F., Guo X. H., Ming X. D. (2022). The decision-making process of offering help in the workplace. *Advances in Psychological Science*.

[4] Billet M. I., Fekken G. C. (2020). The influence of instrumentality in trusting Dark Triad members. *Personality and Individual Differences*.

[5] Calderwood C., Bennett A. A., Gabriel A. S., Trougakos J. P., Dahling J. J. (2018). Too anxious to help? Off-job affective rumination as a linking mechanism between work anxiety and helping. *Journal of Occupational and Organizational Psychology*.

[6] Halbesleben J. R. B., Wheeler A. R. (2015). To invest or not? The role of coworker support and trust in daily reciprocal gain spirals of helping behavior. *Journal of Management*.

[7] Newark D. A., Bohns V. K., Flynn F. J. (2017). A helping hand is hard at work: help-seekers’ underestimation of helpers’ effort. *Organizational Behavior and Human Decision Processes*.

[8] Stea D., Pedersen T., Foss N. J. (2017). The relational antecedents of interpersonal helping: ‘Quantity’, ‘quality’ or both?. *British Journal of Management*.

[9] Wang L., Law K. S., Zhang M. J., Li Y. N., Liang Y. (2019). It’s mine! Psychological ownership of one’s job explains positive and negative workplace outcomes of job engagement. *Journal of Applied Psychology*.

[10] Xie Q., Zhang C. Y., Chen X. P. (2021). Effort reward imbalance and young college teacher’ s anxiety: psychological contract breach as a mediator and over-commitment as a moderator. *Journal of Psychological Science*.

[11] Duran F., Bishopp D., Woodhams J. (2019). Relationships between psychological contract violation, stress and well-being in firefighters. *International Journal of Workplace Health Management*.

[12] Reimann M., Guzy J. (2017). Psychological contract breach and employee health: the relevance of unmet obligations for mental and physical health. *Revista de Psicologia Del Trabajo Y De Las Organizaciones*.

The article "Application of Psychological Contract Theory in Mental Health and Professional Development of University Teachers" was retracted in 2023. Reasons: signs of a paper mill; suspected computer-generated content; unreliable results or conclusions; concerns about the data.

[13] Zhu X. H., Yang C. Q., Tan Q. H., Zou J. W. (2017). Impact of psychological contract breach on individual creativity in university research team. *Science and Technology Management Research*.

[14] Qu R., Janssen O., Shi K. (2015). Transformational leadership and follower creativity: the mediating role of follower relational identification and the moderating role of leader creativity expectations. *The Leadership Quarterly*.

[15] Gardner D. G., Huang G. H., Niu X., Pierce J. L., Lee C. (2015). Organization-based self-esteem, psychological contract fulfillment, and perceived employment opportunities: a test of self-regulatory theory. *Human Resource Management*.

[16] Kiazad K., Seibert S. E., Kraimer M. L. (2014). Psychological contract breach and employee innovation: a conservation of resources perspective. *Journal of Occupational and Organizational Psychology*.

[17] Restubog S. L. D., Zagenczyk T. J., Bordia P., Tang R. L. (2013). When employees behave badly: the roles of contract importance and workplace familism in predicting negative reactions to psychological contract breach. *Journal of Applied Social Psychology*.

[18] Alcover C. M., Rico R., Turnley W. H., Bolino M. C. (2017). Multi-dependence in the formation and development of the distributed psychological contract. *European Journal of Work & Organizational Psychology*.

[19] Arshad R. (2016). Psychological contract violation and turnover intention: do cultural values atter?. *Journal of Managerial Psychology*.

[20] Bal P. M., Smit P. (2012). The older the better! Age-related differences in emotion regulation after psychological contract breach. *Career Development International*.

[21] Qin L. L., Zhang G. J., You L. (2022). Application of CSK encryption algorithm in video synergic command systems. *Journal of Organizational and End User Computing*.

[22] Qin L. L., Yu N. W., Zhao D. H. (2018). Applying the convolutional neural network deep learning technology to behavioural recognition in intelligent video. *Tehnički Vjesnik*.

[23] Siegrist J., Starke D., Chandola T. (2004). The measurement of effort-reward imbalance at work: European comparisons. *Social Science & Medicine*.

[24] Zouaoui S. K., Mohamed F. (2022). The psychological contract is a factor in the success of the entrepreneurial support relationship. *EuroMed J. of Management*.

[25] Siegrist J., Li J. (2016). Associations of extrinsic and intrinsic components of work stress with health: a systematic review of evidence on the effort-reward imbalance model. *International Journal of Environmental Research and Public Health*.

The article "Application of Psychological Contract Theory in Mental Health and Professional Development of University Teachers" was retracted in 2023. Reasons: signs of a paper mill; suspected computer-generated content; unreliable results or conclusions; concerns about the data.

[26] Feuerhahn N., Kühnel J., Kudielka B. M. (2012). Interaction effects of effortreward imbalance and overcommitment on emotional exhaustion and job performance. *International Journal of Stress Management*.

[27] Hewett R., Liefooghe A., Visockaite G., Roongrerngsuke S. (2018). Bullying at work: cognitive appraisal of negative acts, coping, wellbeing, and performance. *Journal of Occupational Health Psychology*.

[28] Rossem R. V. (2018). The times of the faculty:Variations in the length of the workweek of faculty at flemish universities. *Higher Education Studies*.

[29] Anderson R. E. (2008). Implications of the information and knowledge society for education. *International Handbook of Information Technology in Primary and Secondary Education*.

[30] Cao K. Y., Li Z. B. (2016). Psychological contract breach and employee’s voice behavior: the moderating effect of leader member exchange. *Journal of Psychological Science*.

[31] Reimann M. (2016). The moderating role of overcommitment in the relationship between psychological contract breach and employee mental health. *Journal of Occupational Health*.

[32] Zhang X., R Long L., Xia R. (2017). Psychological contract breach and destructive voice behavior:an ego depletion perspective. *Journal of Management Science*.

[33] Meltzer H., Bebbington P., Brugha T., Jenkins R., McManus S., Stansfeld S. (2010). Job insecurity, socio-economic circumstances and depression. *Psychological Medicine*.

[34] Pikhart H., Bobak M., Pajak A. (2004). Psychosocial factors at work and depression in three countries of central and eastern europe. *Social Science & Medicine*.

